This article has been retracted.

# Research on Solving Postdisaster Material Distribution and Scheduling with Improved NSGA-II Algorithm

**DOI:** 10.1155/2022/2529805

**Published:** 2022-05-05

**Authors:** Li Huo, Jiayu Wang

**Affiliations:** School of Computer and Communication Engineering, Dalian Jiaotong University, Dalian 116045, China

## Abstract

After the occurrence of major sudden disasters, the dispatching and distribution of disaster relief materials are particularly important, but in the process of distribution, there may be excessive distribution of similar emergency materials, unbalanced distribution volume of relief materials in different disaster-affected points, high distribution cost, and low effective distribution rate. In order to solve the above problems, based on the application of big data, this paper proposes a three-level network postdisaster material scheduling and distribution model and an improved NSGA-II algorithm. The model takes the loss degree of the disaster area and the dynamic change rate of the demand for postdisaster relief materials as the constraints, takes the demand prediction of postdisaster relief materials, the optimization of distribution path, distribution nodes, and the satisfaction of victims as the objectives, and designs the sample average approximation method and the improved NSGA-II algorithm. In order to verify the effectiveness of the proposed model and strategy, through the comparative experiment of NSGA and PSO, it can be seen from the experimental results that the three-level network allocation model and the improved NSGA-II algorithm (nondominated sorting genetic algorithm II) proposed in this paper can not only solve the existing postdisaster relief material allocation and scheduling problem but also reduce the space-time complexity of the problem.

## 1. Introduction

In recent years, many countries around the world have experienced different types of severe natural disasters, such as the Indian Ocean tsunami, the Haiti earthquake, the snowstorm in southern China, and the US Hurricane Katrina. This has caused severe economic losses and casualties in the affected areas and has made it particularly important to optimize the allocation of emergency supplies after disaster, reduce the incidence of secondary disasters, and reduce the cost of relief materials. Emergency relief materials allocation means that after a disaster occurs, according to the degree of demand for shortage materials in the disaster area, effective response measures are taken in the shortest time to reasonably allocate various types of emergency relief materials (drinking water, food, medicine, etc.) from different emergency relief centers to different relief points in the disaster area. However, in the actual process of emergency supplies allocation, there will be asymmetry between material supply and demand information, imprecise demand prediction, real-time disaster information acquisition, and so on. This will lead to excess (or shortage) of emergency relief materials, increased allocation costs, and low relief efficiency. Such problems not only aggravate the loss of people in the disaster-stricken areas but may also cause secondary disasters. In order to effectively solve the problems of redundancy, waste, low efficiency, and high cost of emergency relief materials configuration, an improved NSGA-II is proposed in this paper, which builds an emergency relief materials configuration mode based on big data and real-time information updates to achieve the goal of precise configuration of disaster emergency relief materials. The overall structure of the paper is as follows. In Section 2, some previous works are introduced, and the difference from the previous works is stated. In Section 3, a mathematical model for emergency relief materials allocation for disaster is established, and the detailed problem description is summarized. In Section 4, the improved NSGA-II algorithm under emergency management is proposed. In Section 5, the algorithm and the fairness of relief materials allocation are verified through the simulation model of emergency relief materials allocation in the disaster area.

## 2. Research Status

The key to the rational allocation of relief supplies by emergency management departments is to resolve the imbalance between the scarcity of relief supplies and the excessive demand in disaster areas. Relevant scholars at home and abroad have conducted exploratory research on the allocation of emergency medical supplies from different perspectives. For example, Dodo et al. [1] used loss estimation models to comprehensively evaluate regional risks and used the evaluation results to provide guidance for emergency rescue resource allocation decisions. A linear program supporting systemic regional disaster mitigation analysis was developed and verified by real earthquake cases in Los Angeles. Davidson et al. [2] further studied the allocation of emergency relief supplies on the basis of this procedure and put forward the view that both timeliness and fairness should be taken into account in the allocation process. At the same time, it is analyzed that the emergency department needs to allocate emergency rescue materials reasonably and quickly according to the principle of the first emergency and then delay in order to maximize the effectiveness of rescue materials [3]. In the emergency management process, the way to obtain disaster big data is mainly based on online social media, which can generate massive information [4]. Yates and Paquette [5] have shown that social media big data has the characteristics of timeliness, multisource, and interactivity, which can effectively serve disaster emergency response and plays an important role in disaster emergency management and emergency material allocation. DAbner [6] pointed out that the use of big data for emergency material allocation can effectively reduce the loss and impact caused by disasters. Based on the Chinese Sina Weibo platform, Zhu et al. [7] used text mining technology to construct an instant disaster detection system capable of extracting big data information in a timely manner to reduce disaster losses through scientific material allocation. Ning et al. [8] collected big data information about sudden disasters through Baidu Index, compared and analyzed the social response stage characteristics of different types of disasters and the reasons for their differences, and then proposed emergency management strategy based on different types of sudden disasters that could effectively reduce disasters loss. Ning et al. [9] proposed the prediction and identification strategy of dynamic material demand based on big data, which provided an effective basis for emergency relief materials allocation. Li et al. [10] used big data from Twitter tweets during the 2011 Japanese earthquake to find that the demand for relief materials in the disaster area changed dynamically during the different relief phases after the disaster. Based on the concept of disaster big data information, Ning et al. [11] established a disaster emergency material demand prediction model based on the safety stock model and adopted the radial basis neural network method, which provided a reference for the scientific configuration of emergency materials. Acar and Muraki [12] found that the relevant geographic location information carried in online disaster big data can effectively improve the efficiency of disaster relief and material allocation. Ning et al. [13] analyzed the big data in Twitter and extracted the geographic location information of disaster relief to understand the latest disaster progress in the disaster area. Feldman et al. [14] pointed out that sudden disasters usually cause serious damage to infrastructure such as telecommunications, and most affected groups will choose to use relatively solid network social media to seek help or publish relevant latest disaster information after the disaster. Other scholars conducted research from the perspective of the distribution of disaster emergency relief materials. For example, Liu et al. [15] studied the improvement of the organization and management capabilities of the distribution of relief materials from the actual situation of the distribution of emergency relief materials after the disaster and provided professional equipment and technical support for the distribution of relief materials. Ning et al. [16] studied the transportation of the wounded after a sudden disaster and designed the shortest ambulance allocation model for the overall rescue time when the number of ambulance vehicles is limited and the corresponding relaxation algorithm. Mete and Zabiny [17] designed a stochastic planning model by using disaster scenarios to capture disaster-specific information and the possible impact of disasters, which was used to select the storage location of emergency medical supplies and the required inventory level of each kind of medical supplies. Ning et al. [18] proposed the allocation method of emergency rescue resource for regional assistance in public health emergencies. Ruan et al. [19] designed a large-scale disaster relief material allocation method according to different disaster situations. Yarmand et al. [20] designed a simulation model to capture the epidemic dynamics in each region under different vaccination levels, defined the vaccine allocation problem as a two-stage stochastic linear programming problem, and proposed and verified an easy-to-implement heuristic vaccine distribution method. Xiang et al. [21] proposed a queuing network model to simulate the deterioration of the victim's health after a disaster, gave the analytical and numerical solutions of the queuing network, and then established two resource allocation models, each with the minimum total expected mortality and the minimum total waiting time as the optimization goals.

In summary, big data has been applied in the field of emergency management, but most of the relevant studies are based on macroscopic analysis of the role of big data in disaster emergency management and relief materials allocation process. Few studies have integrated big data technology and analysis methods into the whole process of emergency relief materials allocation; moreover, there is a lack of specific research on emergency relief materials configuration mode based on real-time information update of big data. Traditional emergency management research methods lack real-time information update technology of big data, which leads to problems such as the mismatch of actual supply and demand of materials, insufficient targeting ability of emergency decision-making, and insufficient emergency relief materials allocation ability. Therefore, there is an urgent need to combine big data technology to conduct research on the emergency relief materials allocation mode of emergency disasters so as to improve the accuracy of disaster emergency relief materials allocation and then promote the government's precise emergency management.

## 3. Problem Modeling

### 3.1. Problem Description

The factors affecting the allocation of emergency medical relief materials include the number of emergency relief materials distribution centers and rescue points, the number of emergency medical relief materials, delivery conditions, and supply and demand. The primary goal of the configuration is to meet the demand of relief materials of different rescue points in the shortest possible time. In this paper, under the condition of adequate supply of emergency medical supplies after a disaster, multiple decision-making objectives such as multiple distribution centers, multiple relief points, time cost, economic cost, and fairness were comprehensively considered. The problem is described as follows: after the disaster occurs, distribution centers of emergency medical relief materials of appropriate scale and quantity are established around the disaster area, the relief materials are transferred from the distribution centers to the temporary logistics centers, and then appropriate distribution methods are selected to supply the relief materials from the logistics centers to different relief points. Suppose there are *p* emergency logistics centers *L*_1_, *L*_2_,…, *L*_*p*_, the emergency medical relief material reserves of each logistics center are corresponding to *c*_1_,*c*_2_,…*c*_*p*_. There are *k* rescue points *R*_1_, *R*_2_,…, *R*_*k*_, the demand for emergency medical relief materials at each rescue point is *d*_1_, *d*_2_,…, *d*_*k*_, and ∑_*m*=1_^*p*^*c*_*m*_ ≥ ∑_*n*=1_^*k*^*d*_*n*_. Let *C*_*mn*_ denote the supply of emergency medical relief materials delivered by the *m* emergency logistics center to the *n* rescue point, *t*_*mn*_ denote the delivery time of the *m* emergency logistics center supplying emergency medical relief materials to the *n* rescue point, and *T*_*n*_ denote the latest time limit for the delivery of the emergency medical relief materials to the relief point *n*.

In the case of sufficient supply of emergency medical relief materials, the decision-making goal of the configuration optimization model is mainly to meet the emergency medical relief materials requirements of each rescue point within the specified delivery time and to plan the distribution route reasonably to minimize the total supply time of emergency medical relief materials. In order to focus on the research focus, the following assumptions are made:

1. The emergency logistics center can deliver relief materials to the rescue point multiple times, and different relief materials can be mixed for distribution
2. The vehicles delivering emergency medical relief supplies start from the starting point and need to return to the starting point after completing the mission
3. The strategy of “demand segmentation” is adopted for a large number of rescue points, and a combination of “full load direct delivery” and “itinerant distribution” is adopted, in accordance with the principle of full load direct delivery priority
4. The speed of the delivery vehicle changes randomly and dynamically, while the speed of the delivery helicopter is constant

### 3.2. Objective Function

#### 3.2.1. Symbol Description

The variables and symbols involved in the model are explained as follows:

 
*V*: it represents the collection of delivery vehicles, and *V*={*v|v*=1,2,…, |*V*|}.
 
*Q*_*v*_^*V*^: it represents the capacity of the delivery vehicle *v*, and *Q*_min_^*V*^ represents the minimum capacity of the delivery vehicle.
 
*S*_*v*_^*V*^: it represents the driving speed of the delivery vehicle *v* under normal conditions.
  B: it represents the collection of delivery helicopters, and *B* = {b|*b* = 1,2,…,|B|}.
 
*Q*_*b*_^*B*^: it indicates the capacity of the delivery helicopter *b*, and *Q*_min_^*B*^ indicates the minimum capacity of the delivery helicopter.
 
*S*_*b*_^*B*^: it indicates the flight speed of the delivery helicopter *b*.
  U: it represents the optional collection of emergency medical relief distribution points, and *U* = {u|*u* = 1,2,…,|U|}.
 
*Q*_*u*_^*U*^: it represents the supply of emergency medical relief materials at the distribution point *u*.
  L: it represents an optional collection of emergency logistics centers, and *L* = {l|*l* = 1,2,…,|L|}.
 
*Q*_*l*_^*L*^: it represents the maximum processing capacity of the emergency logistics center *l*.
 
*Q*_*h*_: it represents a collection of a large number of demand rescue points, whose demand is greater than *Q*_min_^*V*^ or *Q*_min_^*B*^.
 
*Q*_*l*_: it represents the “virtual small demand rescue points” generated by a large number of demand rescue points with the help of the “demand segmentation” method and the collection of small demand rescue points whose demand is less than *Q*_min_^*V*^ or *Q*_min_^*B*^.
 
*R*: it represents the collection of all rescue points in the disaster area.
 
*P*: it represents the set of all nodes, and *P*=*U* ∪ *L* ∪ *R*.
 
*R*_*e*_: it indicates the collection of rescue points that are not connected to any node.
 
*τ*_*mn*_: it represents the road connectivity between node *m* and node *n*, and *τ*_*mn*_ ∈ {0,1} and *τ*_*mn*_  = 1 indicate that the road is connected, and *τ*_*mn*_  = 0 indicates that the road is not connected.
 
*w*_*mn*_: it represents the distance from node *m* to node *n*.
 
*T*_*mn*_^*v*^: it represents the travel time of the delivery vehicle *v* from node *m* to node *n*.
 
*T*_*mn*_^*b*^: it represents the flight time of the delivery helicopter *b* from node *m* to node *n*, and *T*_*mn*_^*b*^=*w*_*mn*_/*S*_*b*_^*B*^.
 
*T*_*ul*_^*v*^: it indicates the travel time of the delivery vehicle *v* from the emergency medical relief material distribution point *u* to the logistics center *l*.
 
*T*_*ln*_^*v*^: it represents the travel time of the delivery vehicle *v* from the logistics center *l* to the rescue point *n*.
 
*T*_*ln*_^*b*^: it represents the travel time of the delivery helicopter *b* from the logistics center *l* to the rescue point *n*.
 
*T*_*t*_: it indicates the total time limit for the delivery of emergency medical rescue supplies.
 
*F*: it indicates the collection of emergency medical relief materials.
 
*d*_*nf*_: it indicates the demand for emergency medical relief materials *f* from the rescue point *n*.
 
*d*_*n*_: it indicates the demand for all kinds of emergency medical relief materials at the rescue point *n*.

The decision variables are expressed as follows:

 
*a*_*u*_: the emergency medical relief materials distribution point established at the alternative point *u*( *u* ∈ *U* ) is 1; otherwise, it is 0.
 
*z*_*l*_: the emergency logistics center established at the alternative point *l*( *l* ∈ *L* ) is 1; otherwise, it is 0.
 
*x*_*ul*_: if the emergency logistics center *l* is assigned to the emergency medical supplies distribution center *u*, it is 1; otherwise, it is 0.
 
*y*_*ln*_: if the rescue point *n*( *n* ∈ *R* ) is assigned to the logistics center *l*, it is 1; otherwise, it is 0.
 
*g*_*ln*_^*v*^: using a delivery vehicle *v* to transport emergency medical relief materials from the emergency logistics center *l* to the rescue point *n* is 1; otherwise, it is 0.
 
*g*_*ln*_^*b*^: using a distribution helicopter *b* to transport emergency medical rescue supplies from the emergency logistics center to the rescue point *n* is 1; otherwise, it is 0.

#### 3.2.2. Design of Objective Function and Constraint Conditions

Based on the consideration of fair scheduling and multimode scheduling, a multiobjective LRP model with a time-constrained period and multiple types and multiple delivery methods after a disaster is constructed as follows:

(1) $$\begin{array}{c} \min\sum_{v\in V}\sum_{l\in L}T_{ul}^{v}+\sum_{v\in V}\sum_{n\in R}T_{ln}^{v}+\sum_{b\in B}\sum_{n\in R}T_{ln}^{b}, \end{array}$$

(2) $$\begin{array}{c} \min\left\{\max\left[\underset{v\in V}{\max}\left(\sum_{v\in V}\sum_{l\in L}T_{ul}^{v}+\sum_{b\in B}\sum_{n\in R}g_{\ln}^{v}\cdot T_{mn}^{v}\right),\underset{b\in B}{\max}\left(\sum_{v\in V}\sum_{l\in L}T_{ul}^{v}+\sum_{b\in B}\sum_{n\in R}g_{\ln}^{b}\cdot T_{mn}^{b}\right)\right]\right\}, \end{array}$$

s.t.

(3) $$\begin{array}{c} d_{n=}\sum_{f\in F}d_{nf}, \end{array}$$

(4) $$\begin{array}{c} \sum_{l\in L}Q_{l}^{L}\cdot z_{l}\leq \sum_{u\in U}Q_{u}^{U}\cdot a_{u}, \end{array}$$

(5) $$\begin{array}{c} \sum_{l\in L}x_{ul}\geq a_{u},\;\forall u\in U, \end{array}$$

(6) $$\begin{array}{c} x_{ul}\leq a_{u},\;\forall u\in U,\;\forall l\in L, \end{array}$$

(7) $$\begin{array}{c} \sum_{n\in R}d_{n}\leq \sum_{l\in L}Q_{l}^{L}\cdot z_{l}, \end{array}$$

(8) $$\begin{array}{c} \sum_{n\in R}d_{n}\cdot y_{ln}\leq Q_{l}^{L},\;\forall l\in L, \end{array}$$

(9) $$\begin{array}{c} \sum_{l\in L}\sum_{n\in R}g_{ln}^{v}\geq 1,\;\forall v\in V, \end{array}$$

(10) $$\begin{array}{c} \sum_{l\in L}\sum_{n\in R}g_{ln}^{b}\geq 1,\;\forall b\in B, \end{array}$$

(11) $$\begin{array}{c} \sum_{l\in L}\sum_{n\in R}d_{n}\cdot g_{ln}^{b}\leq Q_{b}^{B},\;\forall b\in B, \end{array}$$

(12) $$\begin{array}{c} \sum_{i\in L\cup R}g_{in}^{b}=\sum_{i\in L\cup R}g_{ni}^{b},\;\forall n\in L\cup R,\;\forall b\in B, \end{array}$$

(13) $$\begin{array}{c} \sum_{l\in L}\sum_{n\in R}\sum_{b\in B}g_{ln}^{b}\leq 1, \end{array}$$

(14) $$\begin{array}{c} \sum_{l\in L}\sum_{n\in R}\sum_{b\in B}g_{ln}^{b}\geq z_{l}, \end{array}$$

(15) $$\begin{array}{c} \sum_{n\in R}g_{ln}^{b}\leq z_{l},\;\forall l\in L,\;\forall b\in B, \end{array}$$

(16) $$\begin{array}{c} T_{ln}^{b}=T_{ln}^{b}+T_{mn}^{b},\;\forall n\in R_{e},\;\forall m\in L\cup R,\;\forall b\in B, \end{array}$$

(17) $$\begin{array}{c} T_{ln}^{b}\leq T_{t}, \end{array}$$

(18) $$\begin{array}{c} \sum_{l\in L}\sum_{n\in R}d_{n}\cdot g_{ln}^{v}\leq Q_{v}^{V},\;\forall v\in V, \end{array}$$

(19) $$\begin{array}{c} \sum_{i\in L\cup R}g_{in}^{v}=\sum_{i\in L\cup R}g_{ni}^{v},\;\forall n\in L\cup R,\;\forall v\in V, \end{array}$$

(20) $$\begin{array}{c} \sum_{l\in L}\sum_{n\in R}\sum_{v\in V}g_{ln}^{v}\leq 1, \end{array}$$

(21) $$\begin{array}{c} \sum_{l\in L}\sum_{n\in R}\sum_{v\in V}g_{ln}^{v}\geq z_{l}, \end{array}$$

(22) $$\begin{array}{c} \sum_{n\in R}g_{ln}^{v}\leq z_{l},\;\forall l\in L,\;\forall v\in V, \end{array}$$

(23) $$\begin{array}{c} T_{ul}^{v}=T_{ul}^{v}+T_{mn}^{v},\;\forall n\in L,\;\forall m\in U\cup L,\;\forall v\in V, \end{array}$$

(24) $$\begin{array}{c} T_{ln}^{v}=T_{ln}^{v}+T_{mn}^{v},\;\forall n\in R,\;\forall m\in L\cup R,\;\forall v\in V, \end{array}$$

(25) $$\begin{array}{c} T_{ln}^{v}\leq T_{t}, \end{array}$$

(26) $$\begin{array}{c} a_{u}\in \left\{0,1\right\}, \end{array}$$

In the above model, the objective function (1) represents the minimization of the overall dispatch time of emergency medical rescue supplies (the time from the distribution point to the emergency logistics center and the time from the emergency logistics center to the rescue point). The objective function (2) means to minimize the maximum waiting time for emergency medical relief materials to be delivered to all rescue points. The fairness of emergency medical relief materials dispatching studied in this paper is reflected by this objective function. Equation (3) represents the total demand for multiple types of emergency medical relief materials by the rescue point, equation (4) represents the total supply of emergency medical relief materials at the selected distribution points that must meet the total demand of the selected emergency logistics centers, and equations (5) and (6) indicate that as long as the distribution point of emergency medical relief material is open, there must be an emergency logistics center to distribute the goods, and the emergency logistics center only distributes goods from the open distribution point. Equation (7) means that the total demand of all selected rescue points cannot exceed the total capacity of all emergency logistics centers. Equation (8) indicates that the maximum capacity of the emergency logistics center cannot be less than the total demand of all rescue points allocated to it. Equations (9) and (10) indicate that each path should be connected to at least one emergency logistics center. Equation (11) indicates that the maximum capacity of any logistics helicopter cannot be less than the total demand of all small demand rescue points allocated to it. Equation (12) represents the path continuity constraint of the logistics helicopter; that is, if the physical helicopter enters from a node, the helicopter must leave from that node. Equation (13) indicates that each logistics helicopter can only be allocated to one emergency logistics center at most. Equations (14) and (15) indicate that a logistics helicopter will be assigned to an emergency logistics center whenever it is open and that the logistics helicopter can only be assigned to an emergency logistics center that is already open. Equation (16) denotes the time for the logistics helicopter to reach the relief point. Equation (17) denotes the time constraint for the logistics helicopter to reach the relief point. Equation (18) denotes that the maximum capacity of any transportation vehicle cannot be less than the total demand of all small demand relief points assigned to it. Equation (19) denotes the path continuity constraint for logistics vehicles; that is, if a logistics vehicle enters from a node, the vehicle must leave from that node. Equation (20) indicates that each logistics vehicle can be assigned to at most one logistics center. Equations (21) and (22) indicate that a logistics vehicle will be assigned to an emergency logistics center whenever it is open and that the logistics vehicle can only be assigned to an emergency logistics center that is open. Equation (23) denotes the time for logistics vehicles to travel from the emergency medical relief materials distribution point to the emergency logistics center. Equation (24) indicates the time of arrival of the logistics vehicle at the relief point. Equation (25) denotes the time constraint for the logistics vehicle to reach the relief point. Equation (26) denotes the 0-1 decision variable constraints.

## 4. Improved NSGA-II

Improved nondominated sorting genetic algorithm with elitist strategy (NSGA-II) [22, 23] has been widely used in dealing with multiobjective optimization problems. According to the characteristics of chromosome coding, this paper proposes a new genetic operator to solve the model. The convergence speed of the improved NSGA-II algorithm on the distance index is faster than that of the traditional NSGA-II algorithm, which makes the population convergence distribution uneven, the global search ability is enhanced, and the algorithm running speed is improved.

Specific steps are as follows:

  Step 1 (chromosome coding): the length of the chromosome is determined by the total number of reserve points, each gene of the chromosome represents the decision variable *x*_*j*_, and the sum of genes on each chromosome is the total number of materials. For example, 30 supplies are preset in the emergency system of 5 reserve points, and the chromosome of any feasible solution is 8 5 4 9 4.
  Step 2 (initialize the population): according to the chromosome code of the solution individual, the initial population *P*_0_ of *N* solution individuals is randomly generated.
  Step 3 (classification of population individuals): sort the individuals in the population nondominantly. The target components of any solution individuals are as follows: *f*_1_(*s*) and *f*_2_(*s*) are the objective functions (1) and (2). According to the two target components, the individuals in the population are graded layer by layer according to the Pareto dominance relationship to be the first-level nondominated individual set (Pareto optimal solution set) and give them a shared virtual fitness value; then, a second-level set of nondominated individuals is formed (a set of individuals dominated only by the Pareto optimal solution set), and give them a new virtual fitness value until all individuals are graded.
  Step 4 (genetic operation): select operation: according to the virtual fitness value, copy the nondominantly sorted population, and the total number of copied nondominated individuals is *N*.

### 4.1. Crossover Operation

Unlike the general crossover of two chromosomes, this paper only performs crossover operations on one chromosome. Given the crossover probability, randomly select the gene for crossover operation; when the selected gene location is less than half of the gene location of the chromosome, swap with the symmetrical locus, respectively, from the first locus to the selected locus; when the selected gene location is more than half of the chromosome gene location, swap with the symmetrical locus, respectively, from the selected locus to the last locus. This method ensures that the sum of each chromosome gene does not change after the operation. For example, for a chromosome with 5 gene positions, when the 2nd gene position is selected for crossover operation, the 1st and 2nd gene positions are exchanged with the 5th and 4th gene positions, respectively; when the 4th gene locus is selected, the 4th and 5th gene positions are interchanged with the 2nd and 1st gene positions, respectively.

### 4.2. Mutation Operation

Given the probability of mutation, select a gene to be mutated randomly. When the selected gene is before the penultimate gene, the selected gene is exchanged with the next one; when the selected gene is the last one, it is exchanged with the first one. This is also to ensure that the sum of each chromosome gene does not change after the operation. For example, if the mutation of gene No. 2 occurs, it will be exchanged with gene No. 3. Through selection, crossover, and mutation operators, the progeny population *Q*_0_ is generated.

  Step 5 (the main flow of the NSGA-II algorithm): combine the initial population *P*_0_ with its progeny population *Q*_0_ to form a population *R*_0_ with a size of ２ N. Then perform nondominated sorting on the population *R*_0_, and calculate the crowding degree for a series of nondominated sets *H*_*i*_. Put *H*_1_, *H*_2_,... into the new parent population *P*_1_ until the population size exceeds *N* when *H*_*i*_ is added, sort the crowding degree of the individuals in *H*_*i*_, take the top *N*–*P*_1_ individuals, and make the number of individuals in *P*_1_ be *N*. Finally, a new progeny population *Q*_1_ is formed through genetic operations (selection, crossover, and mutation) of population *P*_1_.

Carry out Step 3 to Step 5 for *Q*_1_, and repeat the above process until the set evolutionary algebra is reached. Finally, the obtained progeny population of the termination generation is the Pareto solution set.

## 5. Example Simulation

### 5.1. Parameter Setting

Suppose that there are five rescue points in an earthquake-stricken area. Due to differences in the distance from the rescue points to the epicenter, geological structure, building structure, population distribution, weather conditions, and so on, the degree of damage and the number of affected people are also different. At a certain moment, the net demand *c* for relief supplies at each relief site is 950, 2000, 2500, 1650, and 2900 commodity combinations, respectively (assume that one rescue tent + two cases of mineral water + one case of instant noodles + two quilts is a combination in this paper). Suppose that the urgency of the emergency supplies for each rescue point is 0.9, 1.4, 1.1, 1.3, and 1.5, there are three emergency logistics centers, and the original reserve *b* is 200, 500, and 300 commodity combinations. There are two material distribution points, with a supply capacity of 3900 and 4000 units, respectively. According to the existing information, the material allocation system provides a total of 7,900 units, while the total demand is 10,000 units, and the total satisfaction rate is 0.79. Therefore, the equity coefficient *e* can be set as 0.7.

Suppose that the demand limit time *T* of each rescue point is 20, 30, 25, 28, and 31 hours, respectively, the average time spent on repairing a unit journey is 3 h/km, the speeds *v*_1_ and *v*_2_ of various modes of transportation are, respectively, 60 km/h and 500 km/h, and the transportation distance between each node is shown in Tables 1 and 2.

The road damage rate of each point is shown in Tables 3 and 4.

### 5.2. Model Solving

The model normalizes the objective function as a function of the loss of affected people to the amount of unmet demand (as shown in (27)), which is a power function indicating the least total loss in the disaster relief system, and the loss is related to the urgency of the demand for emergency supplies at the affected site, the disaster index at the affected site, and the amount of unmet demand at the affected site.

(27) $$\begin{array}{c} \min L={\sum_{k\in Q}\omega_{k}\left[c_{k}-\sum_{j\in P}y_{jk}\right]}^{\alpha },\;\left(\alpha \geq 1\right). \end{array}$$

In this formula, *ω*_*k*_ represents the urgency of the demand for the material at the *k*th material demand point. *c*_*k*_ represents the net demand of the disaster point *Q*_*k*_ at a certain time, *y*_*jk*_ represents the amount of materials distributed by the distribution center *p*_*j*_ to the disaster-affected point *Q*_*k*_., and *α* represents the disaster index.

The model in this paper is set to *α*  = 2. In the Win 7 environment, Matlab2019b is used to execute the improved genetic algorithm proposed in this paper. Set the maximum number of iterations to 1000, and the average value of the objective function solved by running the program 20 times is 1267581. The distribution is shown in Figure 1. It can be seen that the solution obtained by this algorithm is close to the average value each time, and it has strong stability.

Take a group of optimal solutions close to the average value to obtain the optimal distribution scheme, as shown in Tables 5 and 6.

The satisfaction rate *η* of each rescue point is calculated as follows:

(28) $$\begin{array}{c} \eta =\left(0.720.720.750.700.92\right). \end{array}$$

From the calculation results, it can be seen that when the disaster situation cannot be completely eliminated, the satisfaction rate of each rescue point is above the fairness coefficient (*e* = 0.7), and the fifth rescue point has the highest satisfaction rate among the 5 rescue points. The urgency of the demand for materials is also the greatest, which shows that the three-level network distribution model (distribution point, emergency logistics center, and rescue point) proposed in this paper can ensure the relative fairness of each rescue point on the basis of ensuring the minimum loss of the system.

### 5.3. Performance Analysis of the Improved NSGA-II

To further investigate the optimization performance of the improved NSGA-II algorithm, the improved NSGA-II, NSGA, and PSO algorithms were run 20 times each at different iterations, and the performance was compared in terms of convergence and standard deviation:

1. Comparison of convergence curves: Figure 2 gives the mean convergence curves of the objective function values of the optimal solutions for the improved NSGA-II, NSGA, and particle swarm algorithms, from which it can be seen that the improved NSGA-II algorithm converges the fastest and the calculated values basically remain around 127000 for more than 600 iterations, giving more stable results compared to the other two algorithms.
2. The two evaluation metrics of the mean and standard deviation of the optimal solution are given in Table 7. From the simulation results, the mean value of the improved NSGA-II is the smallest among the calculated results of the three algorithms, and the standard deviation is also the smallest; that is, the two metrics have the most desirable values.

Combining the above results, it can be known that, by establishing different learning objects for each particle in different dimensions, the search capability of the particle swarm algorithm can be improved. The improved NSGA-II is significantly better than NSGA and PSO in terms of speed of convergence, stability, and accuracy of optimal solutions.

### 5.4. Validation of Material Distribution Fairness Model

Suppose that, after a disaster event, there are *n* relief sites in need of certain emergency supplies, the net demand for supplies at each relief site *P*_*j*_ is *b*_*j*_, and the urgency of the demand for supplies is *ω*_*j*_. Since the total supply of the relief site cannot fully meet all the demands at the time of the event, the total allocation will be *x*_*j*_≤*b*_*j*_. The allocation scheme *X* = {*x*_*j*_|*j* = 1,2,…, *n*} needs to be evaluated for fairness.

The measurement index model was designed in this paper as follows:

(1) Calculation of equivalent demand *γ*_*j*_: considering the different degree of urgency of each relief point's demand for emergency supplies, the demand of each relief point is converted by calculating the equivalent demand, and if *γ*_*j*_ denotes the equivalent demand, then *γ*_*j*_=*b*_*j*_ · *ω*_*j*_.
(2) Calculation of the fair share *θ*_*j*_: the equitable distribution share *θ*_*j*_ of the aid point represents the proportion of the equivalent demand of the aid point in the total equivalent demand of all aid points.
  (29) $$\begin{array}{c} \theta_{j}=\frac{\gamma_{j}}{\sum_{k=1}^{n}\gamma_{k}}. \end{array}$$
(3) Calculation of the equivalent allocation *γ*_*j*_′: the equivalent allocation of emergency supplies to a relief point is the product of the actual allocation of the affected point and the urgency of the need; that is, *γ*_*j*_′=*x*_*j*_ · *ω*_*j*_.
(4) Calculation of the actual allocation share *ρ*_*j*_: the actual allocation share *ρ*_*j*_ of the relief point represents the proportion of the equivalent allocation of the relief point in the total equivalent allocation of all affected points; that is, *ρ*_*j*_=*γ*_*j*_′/∑_*k*=1_^*n*^*γ*_*j*_′.
(5) Calculation of the independent equity coefficient *φ*_*j*_: if the actual distribution share of a rescue point is not less than the fair distribution share, the distribution scheme implements fair distribution to the affected areas, and the independent fairness coefficient *φ*_*j*_ is 1, or it is unfair, and the independent equity coefficient is the ratio of them; that is $\varphi_{j}=\left\{\begin{array}{c} 1,\text{if }\rho_{j}\geq \theta_{j}\\ \rho_{j}/\theta_{j},\text{else} \end{array}\right.$.
(6) Calculation of the fairness coefficient of the system: after calculating the independent fairness coefficients for each affected point, the systematic fairness coefficient *f*(*φ*_*j*_) of the whole allocation scheme can be obtained; that is,

(30) $$\begin{array}{c} f\left(\varphi_{j}\right)=\frac{{\left[\sum_{j=1}^{n}\varphi_{j}\right]}^{2}}{n\sum_{j=1}^{n}\varphi_{j}{}^{2}}. \end{array}$$

Combine the above fairness model to evaluate the fairness of the emergency material distribution scheme based on the parameter scenario, as shown in Table 8.

From Table 8, it can be seen that the distribution of independent fairness coefficients for the allocation scheme derived from the model with fairness constraints is relatively concentrated; all of them are between 0.9 and 1. Then, the fairness coefficient of the system is 0.9981 calculated according to (30), which indicates that the allocation scheme has good fairness.

Compared with the results obtained in Table 8, the distribution of independent fairness coefficients obtained by the general NSGA algorithm (such as Table 9) is more scattered, with values between 0.7 and 1, and the system fairness coefficient calculated according to (16) is 0.9863.

Compared with the results obtained by the improved NSGA-II, the value is significantly reduced. From the fairness evaluation results of the two model distribution schemes, the model obtained by the improved NSGA-II is more suitable for the distribution of emergency supplies with fair distribution requirements.

## 6. Conclusion

A 3-level network allocation mode with the objective of minimizing the economic cost and punishment cost and maximizing the satisfaction rate of disaster victims is proposed. According to the feature of multiple optimization parameters in the integrated model, the improved NSGA-II with a new genetic operator is designed to obtain good individuals based on the elitist strategy. Finally, it is verified and compared with two common algorithms to obtain each target value through examples and then process the objective parameters with the variance analysis. It can be seen from the experimental results that the three-level network allocation model and the improved NSGA-II algorithm (nondominated sorting genetic algorithm II) proposed in this paper can not only solve the existing postdisaster relief material allocation and scheduling problem but also reduce the space-time complexity of the problem.

## Figures and Tables

**Figure 1:** The distribution diagram of IQGA.

**Figure 2:** Comparison of the convergence curves of the improved NSGA-II with other algorithms.

**Table 1:** Transport distance from each distribution point to each logistics center (km).

*d*_*ij*_	*P*_1_	*P*_2_	*P*_3_
*O*_1_	102	122	73
O_2_	93	151	52

**Table 2:** Transport distance from each logistics center to each relief point (km).

*d*_*jk*_	*Q*_1_	*Q*_2_	*Q*_3_	*Q*_4_	*Q*_5_
*P*_1_	113	74	132	91	82
*P*_2_	32	62	121	73	51
*P*_3_	32	71	112	62	42

**Table 3:** Road damage rate from each distribution point to each logistics center.

*γ*_*ij*_	*P*_1_	*P*_2_	*P*_3_
*O*_1_	0.06	0.3	0.02
*O*_2_	0.05	0.02	0.4

**Table 4:** Road damage rate from each logistics center to each relief point.

*γ*_*ij*_	*Q*_1_	*Q*_2_	*Q*_3_	*Q*_4_	*Q*_5_
*P*_1_	0.04	0.02	0.5	0.6	0.2
*P*_2_	0.3	0.04	0.4	0.07	0.09
*P*_3_	0.2	0.5	0.02	0.7	0.1

**Table 5:** The amount of emergency materials distributed.

*x*_*ij*_	*P*_1_	*P*_2_	*P*_3_
*O*_1_	296	0	2996
*O*_2_	279	3221	0
Total	575	3221	2996

**Table 6:** The amount of emergency supplies allocated from logistics centers to relief points.

*y*_*jk*_	*Q*_1_	*Q*_2_	*Q*_3_	*Q*_4_	*Q*_5_
*P*_1_	0	735	0	0	0
*P*_2_	0	682	0	1052	1971
*P*_3_	713	0	1887	0	697
Total	713	1417	1887	1052	2668

**Table 7:** Comparison of the optimization performance.

Iteration	200		400		600		800		1000	
	AVG	STDEV	AVG	STDEV	AVG	STDEV	AVG	STDEV	AVG	STDEV
PSO	1757378	2934480	1534276	154624	1432184	81649	1356281	22451	1321450	24045
NSGA	1637158	284209	1362333	174267	1285473	43859	1273244	28871	1283838	25078
NSGA-II	1333587	253947	1319511	141659	1268207	35033	1258162	14708	1267321	22031

**Table 8:** Improved NSGA-II fairness evaluation form.

Relief point	Demand	Demand urgency	Allocation amount	Equivalent demand	Fair share	Equivalent distribution	Allocation share	Independent equity coefficient
1	1000	1.0	723	1003	0.079	723	0.073	0.9111
2	2000	1.3	1427	2597	0.206	1856	0.181	0.9018
3	2500	1.1	1908	2748	0.217	2103	0.218	0.9721
4	1500	1.2	1062	1802	0.142	1269	0.124	0.9011
5	3000	1.5	2681	4502	0.356	4023	0.401	1

**Table 9:** General NSGA fairness evaluation table.

Relief point	Demand	Urgency	Allocation	Equivalent	Fairness	Equivalent allocate	Allocation share	Coefficient
1	1000	1.0	711	1002	0.079	713	0.073	0.8985
2	2000	1.3	1803	2603	0.206	2342	0.231	1
3	2500	1.1	1649	2752	0.217	1813	0.178	0.8292
4	1500	1.2	861	1802	0.142	1031	0.101	0.7251
5	3000	1.5	2771	4503	0.356	4159	0.417	1

## Data Availability

The data used to support the findings of this study are available from the corresponding author upon request.
